# Research on Emotion Recognition of EEG Signal Based on Convolutional Neural Networks and High-Order Cross-Analysis

This article has been retracted.

**DOI:** 10.1155/2022/6238172

**Published:** 2022-02-15

**Authors:** Chengcheng Fan, Xiang Liu, Xuelin Gu, Liang Zhou, Xiaoou Li

**Affiliations:** ^1^Shanghai University of Medicine & Health Science, School of Medical Instrument, 257 Tianxiong Road, Pudong New District, Shanghai 201318, China; ^2^Department of Automation, School of Mechatronics Engineering and Automation, Key Laboratory of Power Station Automation Technology, Shanghai University, 333 Nanchen Road, Shanghai 200072, China; ^3^Weihai Municipal Hospital, 70 Heping Road, Huanchui District, Weihai 264200, China

## Abstract

Emotion recognition means the automatic identification of a human's emotional state by obtaining his/her physiological or nonphysiological signals. The EEG-based method is an effective mechanism, which is commonly used for the recognition of emotions in real environments. In this paper, the convolutional neural network is used to classify the EEG signal into three and four emotional states under the DEAP dataset, which is defined as a Database for Emotion Analysis using physiological signals. For this purpose, a high-order cross-feature sample is extracted to recognize the emotional state with a single channel. A seven-layer convolutional neural network is used to classify the 32-channel EEG signal, and the average accuracy of four and three emotional states is 65% and 58.62%. The single-channel high-order cross-sample is classified with convolutional neural networks, and the average accuracy of four emotional states is 43.5%. Among all the channels related to emotion recognition, the F4 channel gets the best classification accuracy of 44.25%, and the average accuracy of the even number channel is higher than the odd number channel. The proposed method provides a basis for the real-time application of EEG-based emotion recognition.

## 1. Introduction

Emotion is a state that synthesizes a human's feelings, thoughts, and behaviors. It includes the psychological response to external or oneself stimulation and the physiological reaction accompanied by this psychological reaction. The role of emotional appearance exists in human's daily work and life [1]. In the medical area, if the emotional state of the patient is detected, especially those patients with expression disorders, doctors can make different medical measures according to patients' emotions and improve the quality of medical care [2].

Emotion is a physiological state produced by comprehensive senses, thoughts, and behaviors [3]. Emotions are reflected in the brain activity which is accompanied by a corresponding electroencephalogram [4]. On the other hand, human emotions are complex; in particular, hidden emotional experiences are easy to conceal by various appearances. As the whole expression of brain activity is produced in the central nervous system, EEG signals cannot be easily regulated by the corresponding person, and the emotion decoding based on EEG signals can analyze the emotion from the most fundamental physiological signal [5].

Artificial Intelligence (AI) is an emerging research domain which is growing very fast specifically to form a bridge between technology and its adoption in solving real-world problems specifically those related to the health sector. For this purpose, Convolution Neural Network (CNN), which is an important aspect of traditional artificial intelligence, is utilized in resolving various real-world problems specifically in the healthcare domain. Therefore, in this paper, we have utilized the potentials of the convolution neural networks in resolving the aforementioned issue, that is, emotion recognition of EEG signals in the healthcare sector. To realize this, we have used experimental data, where patients are divided into two different groups. The main scientific contribution of this paper is given as follows.

- A convolution neural network-enabled emotion decoding is specifically based on electroencephalogram signal
- A sophisticated mechanism or model is designed which is used for the extraction of emotion-related features from EEG signals
- Convolution neural network along with an appropriate classification algorithm is used to classify the EEG emotion features in the healthcare domain

The remaining sections of this paper are arranged as follows.

In the subsequent section, the proposed convolutional neural networks enabled mechanism is presented where the feature extraction method is explained. In Section 3, various experimental results are described and explained along with the effectiveness of the proposed CNN-enabled method. A sophisticated discussion section is provided where a problem statement along with a suitable solution is provided. Finally, concluding remarks are provided.

## 2. Materials and Methods

### 2.1. Convolutional Neural Networks

With the intensive study of deep learning algorithms, the application of the proposed algorithm or mechanism in target recognition is becoming widespread especially in the image recognition area [6]. Moreover, deep learning algorithm has a natural advantage in multiclassification recognition. As long as a certain amount of data exists, a deep learning network can be established and trained completely for multiclassification recognition [7].

Compared with other deep learning decoding algorithms, a convolutional neural network (convolutional neural network, CNN) directly uses less preprocessing procedure for target block convolutional pooling. Filters in traditional network algorithms are mostly designed manually, but the advantage for CNN is the independence of the prior knowledge features. CNN has a good effect on image recognition and natural language processing [8]. Convolutional networks are inspired by biological processes because the connection patterns between neurons are similar to those in the animal visual cortex [9]. Individual cortical neurons respond to external stimulation only in areas known as receptive fields. The senses of different neurons overlap to cover the entire field. The application of CNN in image recognition is very mature in computer science. The image can be recognized as a matrix containing pixels, and the EEG signal can also be recognized as a multichannel digital signal, which is similar to a special image. Therefore, EEG signals have great potential to be classified and recognized by CNN.

The CNN is the same as the other classical neural network, which consists of an input layer, multiple hidden layers, and an output layer. The CNN structure is composed of an input layer and a two convolutional layer and a pooling layer, a full connection layer, and an output layer. The network topology diagram is shown in Figure 1.

The hidden layer of CNN is usually composed of convolution layer, pooling layer, full connection layer, and normalization layer. In fact, in the convolutional process of the hidden layer network, it is a kind of convolution which is a kind of correlation rather than a positive integer convolution in mathematical meaning. This only makes sense for the indexes in the matrix which is the position of weights. The function of the convolution layer is to extract various features of the target and the role of the pooling layer is to abstract the original feature signal; thus, it can greatly reduce the number of training parameters and reduce the degree of model overfitting at the same time [10–12].

#### 2.1.1. Convolution

The convolution layer applies the convolution operation to the input and passes the result to the next layer. Convolution simulates the response of individual neurons to visual stimulation [13]. Each of the convolutional neurons processes only the data of its receiving field. Although fully connected feedforward neural networks can be used to learn features and classify data, it is impractical to apply this architecture to images. Because of the large input size associated with the image, each pixel is a dependent variable, so even in a shallow (relative to deep) architecture, a very large number of neurons are needed. For example, the fully connected layer of the image 100*∗*100 has a weight of 10,000 for each neuron in the second layer. Convolution provides a solution to this problem for it reduces the number of available parameters and optimizes the network. For example, regardless of the size of the image, a plain area of 5*∗*5 (each area has the same shared weight) requires only 25 parameters to learn. In this way, the problem of disappearing or exploding gradient in the training of traditional multilayer neural networks can be solved by using backpropagation.

In the forward propagation phase, the layer *l* is assumed to be a convolution layer; the layer *l* − 1 is a pooling layer. Then, the formula for layer *l* can be listed as follows:

(1) $$\begin{array}{c} x_{j}^{l}=f\left[\sum_{i\in M_{j}}x_{i}^{l-1}*k_{ij}^{l}+b_{j}^{l}\right]. \end{array}$$

The left part *x*_*j*_^*l*^ demonstrates the *j* feature pattern of layer *l*. The right part demonstrates the convolution and summation of all the connection feature patterns *x*_*i*_^*l*−1^ of *l* − 1 layer and the *j* convolutional kernel *k*_*ij*_^*l*^ of layer *l*, and then, a bias parameter is added for the final activation function *f*[·]. The activation function is called Relu(Rectified Linear Units, Relu). The equation is listed as follows:

(2) $$\begin{array}{c} f\left(x\right)=max\left(0,x\right). \end{array}$$

For the negative value of the input, the output is all zero; for the positive input, the output keeps the original value. It increases the nonlinear characteristics of the decision function and the whole network without affecting the acceptance field of the convolution layer.

The convolution layer is the core component of CNN. The parameters of the layer consist of a set of filters (or kernels) that have smaller acceptance fields but extend to the full depth of the input area. In the forward process, each filter is involved in the width and height of the input kernel, calculates the dot result between the filter entry and the input, and generates the two-dimensional activation diagram of the filter. Therefore, the network learns to activate the filter when it detects a particular type of feature at a certain spatial location in the input. The activation diagrams of all filters stacked along the depth dimension form the full output of the convolution layer. Therefore, each item in the output field can also be interpreted as the output of the neuron, which examines the neuron domain in the input and shares the parameters of the neurons in the same activation graph. CNN shares weights in the convolution layer, which means that each acceptance area in the layer uses the same filter, which reduces memory occupation and improves performance [14].

#### 2.1.2. Pooling

The pooling layer is also known as the downsampling layer; the goal of this layer is to reduce the feature pattern. The pooling operation is independent of each layer; the dimension is generally 2*∗*2 or 3*∗*3.

Another important concept of CNN is aggregation, which is a nonlinear downsampling method. There are several nonlinear functions to implement the pooling, from which the max-pooling is the most common method. It divides the input image into a set of nonoverlapping rectangles and outputs the maximum value for each subregion. Intuition is that the location extraction of features is not more important than the rough location of other features. The pooling layer is used to gradually reduce the space size of the representation to reduce the number of parameters and computation complexity in the network and therefore to control the overfitting phenomenon. It is common to periodically insert pooling layers between successive convolution layers in CNN architecture. The aggregation operation provides another form of interpretation invariance.

The pooling layer runs independently on each layer of the input and adjusts the size spatially. The most common form is a convergent layer of a 2*∗*2 size filter, giving up 75% activation along the width and height of each input deep layer with two downsampled stripes of 2. In this case, each maximum operation exceeds 4 digits. The deep dimension remains the same.

#### 2.1.3. High-Order Cross-Analysis

Almost all observed time-series signals show local and global up-and-down motions over time. This behavior is found in finite zero mean vibration {*Z*_*t*_, t=1,2,…,N}; zero level can be represented by a zero-crossing count. In general, when a filter is applied to a time series, its vibration will be changed, so its zero-crossing count will also change.

In this view, the following iteration processes can be assumed: filtering the time series and counting the zeros in the filtered time series; applying another filter to the original time series, the zero-crossing and counting are observed again, and the filtered zero count sequence of the original time series can be obtained by iterating the filtering and counting process.

This sequence becomes the high-order crossing (HOC) sequence of the time series [15]. When a particular filter sequence is applied to a time series, a corresponding zero-crossing count sequence is obtained, thus producing a so-called HOC sequence. According to the required spectral and resolution analysis, many different types of HOC sequences can be constructed by appropriate filter design. Δ is defined as backward difference factor; the backward difference operator of time series can be defined as

(3) $$\begin{array}{c} \Delta Z_{t}=Z_{t}-Z_{t-1}. \end{array}$$

Backward difference factor Δ is a high-pass filter, if we define the following high-pass filter sequence:

(4) $$\begin{array}{c} {ℑ}_{k}\equiv \Delta^{k-1},k=1,2,3,\ldots . \end{array}$$

When *k*=1, it is the original backward difference factor operation. According to the operator defined by formula (4), we can get the HOC sequence as follows according to the backward difference formula:

(5) $$\begin{array}{c} D_{k}=NZC\left\{\left(Z_{t}\right)\right\},k=1,2,3,\ldots ;t=1,\ldots ,N{ℑ}_{k}. \end{array}$$

*NNZC*{·} represents the zero-crossing count of a sequence. The *ℑ*_*k*_(*Z*_*t*_) operator is shown as follows:

(6) $$\begin{array}{c} \Delta^{k-1}Z_{t}=\sum_{j=1}^{k}\frac{\left(k-1\right)!}{\left(j-1\right)!\left(k-j\right)!}{\left(-1\right)}^{j-1}Z_{t-j+1}. \end{array}$$

In practice, we have only limited time series, and each difference will lose the observation result. Therefore, in order to avoid this influence, we must index the data by moving to the right; that is, for the evaluation of *k* HOC, we should give the index *t* = 1 to the *k*-th or rely on later observation.

For the convenience of zero-counting, the binary time sequence *X*_*t*_(*k*) is defined as

(7) $$\begin{array}{c} X_{t}\left(k\right)=\left\{\begin{array}{cc} 1, & {ℑ}_{k}\left(Z_{t}\right)\geq 0,\\ 0, & {ℑ}_{k}\left(Z_{t}\right)<0, \end{array}\right.k=1,2,3,\ldots ;t=1,\ldots ,N. \end{array}$$

So the calculation of *X*_*t*_(*k*) zero-crossing count can get the *ℑ*_*k*_(*Z*_*t*_) zero-crossing *D*_*k*_.

(8) $$\begin{array}{c} D_{k}=\sum_{t=2}^{N}{\left[X_{t}\left(k\right)-X_{t-1}\left(k\right)\right]}^{2} \end{array}$$

In the limited time series, *D*_*k*+1_ ≥ *D*_*k*_ − 1 [16]. And when *k* increases, the variation of HOC sequences becomes smaller and smaller; that is to say, when *k* is increased to a certain degree, *D*_*k*+1_ and *D*_*k*_ tend to be equal. In this paper, HOC sequence is used as the feature of EEG-related emotion elements as

(9) $$\begin{array}{c} FV_{\text{HOC}}=\left[D_{1},D_{2},\ldots ,D_{L}\right],\;1<L\leq J, \end{array}$$

where *J* is the highest order of the HOC sequence.

## 3. Description of the Experimental Data

This experiment utilizes the International EEG emotion database DEAP (DEAP: A Database for Emotion Analysis using Physiological Signals). DEAP is a multimodal data which is set to analyze the emotional state of human beings. Electroencephalogram and peripheral physiological signals were recorded in 32 subjects. Each subject watched a 40-minute excerpt of the music video and rated each video according to arousal, valence, like/dislike, advantage, and the familiar degree [17]. DEAP had 32 subjects in the experiment, each subject watched a 60-second video, and the first three seconds were the time for the subjects to calm down. The length of each trial is 63 seconds, and the emotion EEG data is collected when viewing the film 60 seconds later. One session has 40 trials. The collected EEG data is preprocessed with a 4∼45 Hz band-pass filter.

## 4. Experiment and Results

### 4.1. Research on Four Categories of EEG Emotion Decoding Based on CNN (Happy, Angry, Sad, and Relaxed)

#### 4.1.1. Research on Four Categories of Emotion Decoding Based on the 32 Channel

Each subject does a 40-session experiment, each session has 40 trials of emotional movies, and the time for the movie is 60 seconds for recording EEG signal with a sampling frequency of 128 Hz. Take the time window length of 0.5 s to calculate the emotional state, so the sample number of each subject is Nsample_each_person_=40 × 60 ÷ 0.5=4800. So, the sample is in the form of 32 × 64; we segment the data to 32 × 32 for calculation. The total sampling number obtained from four different subjects is *N*sum=4800 × 4 × 2=38400.

The four categories of emotion labels were obtained according to the two factors of valence and arouse in the two-dimensional model of Russel emotion. Both dimensions were evaluated in the DEAP database based on the self-assessment model (SAM). The SAM model is shown in the following Figure 2.

The subjects were evaluated objectively on the basis of 1 to 9 on two dimensions after watching emotional videos. Starting with the middle number of 5, you can get four categories of emotion labels as shown in Figure 3.

Therefore, in the DEAP dataset, we can get four types of emotion labels: happy, angry, sad, and relaxed. The total sampling number of four groups of subjects was 38400, and the sampling number of the four categories of emotion labels was shown in Table 1.

In this experiment, the seven layers of the convolutional neural network are used: input layer, convolution layer 1, pool layer 1, convolution layer 2, pool layer 2, full connection layer, and output layer. The convolutional kernel is 9 × 9, one training module consists of 100 groups of data, and learning efficiency is 1. A fourfold cross-validation method was used for 20000 sets of sampling data. The mean error of the model is shown in Figure 4.

The correct rate of emotion decoding in four experiments is shown in Figure 5.

The average accuracy of the 5000 groups of the test sample was 63%, 64%, 65%, and 65%, respectively. The average accuracy of the four groups of experimental data of happiness, anger, sadness, and relaxation was 64.25% in the DEAP International emotion EEG Database. This resolution is far greater than the random accuracy of 25%. So, we can get the result that a convolutional neural network can recognize EEG data and classify the emotion state well.

#### 4.1.2. Research on the Four Categories of Emotion Decoding Based on a 10-Channel EEG Signal

Over the past few years, researchers have focused on finding chief frequencies and channels for EEG-based emotion decoding in different ways. EEG emotion recognition based on a small number of channels is an important topic in the application of emotion recognition. Using a small number of channels can reduce the recognition time and reduce the influence of useless channels on the recognition state, which could play a positive role in the establishment of the model.

Bos et al.. proved that *Fpz*, *F*3, and *F*4 channels are the most appropriate electrode position for measuring the value of emotion effects according to the valence and arouse classification research [18].

Combined with existing research results, Valenzi et al. use *AF*3, *AF*4, *F*3, *F*4, *F*7, *F*8, *T*7, and *T*8 channels to get an 87.5% average accuracy [16]. However, how to select critical channels and how to evaluate the selected electrodes have not been fully studied.

This paper gathers the emotion-related channels in the existing literature: *AF*3, *AF*4, *F*3, *F*4, *F*7, *F*8, *T*7, *T*8, *FP*1, and *FP*2 channels are used to classify the 4 categories of happy, angry, sad, and relaxed using CNN. The EEG experimental module includes 10 × 32, 9 × 9 kernel, and 100 data for a training module; the learning efficiency is 1. 20000 groups of sampling data were tested by 4-time cross-validation. The experiment result is listed in Figure 6.

Figure 7 shows the CNN training result of 40, 60, 80, and 100 iterations; the corresponding decoding accuracy of Figure 6 is 53.74%, 54.26%, 54.36%, and 54.55%. Compared with the 32-channel classification accuracy of 63%, 64%, 65%, and 65%, the correct rate is 10% lower, but the decoding time is fewer. The time of each experiment is 28 seconds for the 32-channel model building process but 6.5 seconds for the 10-channel experiment; the time for each experiment model establishment is 21.5 seconds fewer. For example, the 40-iteration CNN model establishes the time reduction 860 s, which is very important in practical applications.

### 4.2. Research on Three Categories of EEG Emotion Recognition Based on CNN (Happy, Calm, and Sad)

In this section, we discuss the implementation of CNN to categorize three emotions of happy, calm, and sad in DEAP. Classification criteria for emotional labels are according to the given valence dimension. The specific classification is shown in Table 2.

The EEG signals in three emotional states of happiness, calmness, and sadness are shown in Figure 8.

Take the time window length of 0.5 seconds to calculate the emotional state; the number of samples obtained by each subject was Nsample_each_person_=40 × 60 ÷ 0.5=4800. So, the sample form is 32 × 64, For later calculation, we split the data into the form of 32 × 32. The total number of samples obtained from four different subjects is Nsum=4800 × 4 × 2=38400. 30000 groups of samples were taken to train the CNN model, and the remaining 8400 groups of samples were used to test the accuracy of the three categories of emotion classification.

The number of iterations of training means that 30000 groups of training data are trained in the cycle, and 8 times of training means that after training 30000 groups of training data, 30000 groups of sample data will continue to be input into the model and adjust the model so that the model can be adjusted 8 times. As is shown in Figure 9, the model error is more than 0.2 when training for 8 or 10 iterations; then, it continues to train 20 iterations. After 30 times, the model error can be lower than 0.2; then, the model error can maintain a steady state after 20–30 times of iterations. According to 4 times of 8400 test samples, the classification accuracy is 0.5706, 0.5862, 0.5939, and 0.5941, as shown in Figure 10.

From Figure 10, the model iterations ranging from 8 to 20 with the accuracy for happy, calm, and sad are increasing correspondingly. It is not obvious of the accuracy increase for 20–30 times of iterations. The four categories of iteration models using CNN model accuracy based on EEG are 0.5706, 0.5862, 0.5939, and 0.5941; the average accuracy is 58.62% which is better than the random accuracy of 33.33%.

### 4.3. Single Channel Emotion Decoding Based on HOC Feature of DEAP Database

Emotion decoding is an important direction of artificial intelligence in the future. The research of emotion decoding based on a single channel is a necessary way in the application of emotion decoding. There are few researches on emotion decoding based on a single channel; because of the simple architecture and low dimension of the EEG HOC feature, it is appropriate to research the single-channel emotion decoding.

The main research of this section is about the single-channel emotion decoding based on DEAP EEG HOC features. A four-second HOC feature of EEG data with a sampling frequency of 128 Hz was selected as a sample for emotion decoding. First, the highest-order HOC features within 4 seconds are found which represents the *J* value in equation (9). This *J* value represents the highest dimension of the HOC feature. Second, the HOC feature data labeled happy and sad from the *F*3 channel is extracted. The *K* value from equation (9) ranges from 8 to 13 to find the HOC feature with the highest dimension. The result is shown in Figure 11.

From Figures 11 and 12, no matter the happy label or sad label in four seconds of EEG data, when *k* = 10, the HOC sequence reaches the maximum and remains steady without the influence of *k* value increase. It is shown that the order of the HOC sequence of 4 s EEG data based on backward difference operator is 10. That means the following HOC feature dimension is 10.

The dataset used in this method is 20 packets from the DEAP. Each packet contains 40 groups of experiments lasting for 63 seconds, in which the first 3 s are ready for the experiment in a calm state. The later 60 seconds were EEG data with specific affective factors, and the sampling frequency was 128 Hz. Taking 4 seconds of EEG emotion data as an experimental judgment, we can get 12000 groups of labeled experimental samples.

According to the previous study, the 10 electrodes with the greater affective relationship were selected as follows: *AF*3, *AF*4, *F*3, *F*4, *F*7, *F*8, *T*7, *T*8, *FP*1, and *FP*2 located in the symmetrical position of the left and right brain. The 10-order HOC sequence of the backward differential operator with 10 electrodes was extracted as an EEG emotion feature, and the convolutional neural network was used to classify the emotion features into four categories: happy, angry, sad, and calm. 10000 groups of samples were randomly selected for training and 2000 groups of samples were tested. The classification accuracy is shown in Figure 13.

It can be seen from the above image that the average accuracy of the four categories of emotion classification based on the HOC sequence features of EEG signals is 43.5%. Within the 10 electrodes, the classification results of *AF*3, *AF*4, *F*3, *F*4, and *FP*2 are better than the other 5 electrodes. Second, we can find that the classification accuracy of even position electrodes is higher than that of odd position electrodes; for example, the classification accuracy of even position electrodes *F*4 is higher than that of odd position electrodes *F*3. The results showed that the right hemisphere had an advantage in emotion recognition, and the expression of emotion and the control of related behaviors occurred mainly in the right hemisphere. It is consistent with the idea that the right brain is responsible for emotion perception.

## 5. Conclusion and Discussion

This paper introduces the research of EEG emotion decoding based on a convolutional neural network and high-order cross-analysis. Convolution is equivalent to a filter. The EEG module is filtered by a convolution kernel to obtain the convolution layer. The pooling layer is a further abstraction of the convolution layer. In this experiment, the maximum pooling method is used to downsample the convolution layer, which greatly reduces the parameters and further reduces the training time. Four groups of experimental data in DEAP were used to test the convolutional neural network. 20000 groups of samples are used to train 10, 20, 30, and 40 iterations with the method of 4 times of cross-validation, so the corresponding happy, angry, sad, and calm decoding accuracy is 63%, 64%, 65%, and 65%; the average correct rate is 64.25% which is far greater than the opportunity correct rate of 25%. Therefore, the convolution neural network can be applied to the multiple classification of EEG emotion recognition. Then, the experiment of happy, calm, and sad classification of EEG signals based on CNN classification network is explored. The difference with the four categories is that four categories of labels determine two dimensions of valence and arousal using Russel's two-dimensional model and the three categories only use the effect value dimension 3 to classify the three kinds of labels. The average classification accuracy is 58.62% after 8 iterations, 10 iterations, 20 iterations, and 30 iterations of training. Finally, emotion recognition based on a single channel is discussed, ten channels that are most relevant to emotion are selected, HOC feature samples of 10 channels with a 4-second window length are extracted from the international emotional database DEAP, the convolutional neural network is implemented to classify the happy, angry, sad, and relaxed labels, and the average correct rate is 43.5%. Channel *F*4 has the highest correct rate of 44.25%; the classification accuracy of even-numbered channels is higher than that of odd channels. The right hemisphere is predominant in emotion recognition, and the control of emotion expression and related behaviors occurs mainly in the right hemisphere, which is the even-numbered channel.

## Figures and Tables

**Figure 1:** CNN topology diagram.

**Figure 2:** SAM self-assessment model.

**Figure 3:** Four categories label.

**Figure 4:** Mean error of four categories of emotion decoding training models based on CNN.

**Figure 5:** CNN decoding accuracy using 32 channels.

**Figure 6:** Mean error for 10 channels training based on CNN.

**Figure 7:** CNN training accuracy of emotion decoding using 10 channels.

**Figure 8:** EEG signals for happy, calm, and sad.

**Figure 9:** Mean error for valence dimension training based on CNN.

**Figure 10:** CNN decoding accuracy under valence dimension.

**Figure 11:** HOC order of 4 s happy EEG under DEAP dataset.

**Figure 12:** HOC order of 4 s sad EEG under DEAP dataset.

**Figure 13:** SAE decoding accuracy under the single channel.

**Table 1:** Sampling number of four-category emotions.

Emotion	Happy	Angry	Sad	Relaxed
Samples	10320	6960	1760	9360

**Table 2:** Valence dimension emotion labeling 3 categories.

Valence	Valence ≤ 3	3 < valence ≤ 6	6 < valence ≤ 9
Emotion state	Sad	Calm	Happy
Label	[1; 0; 0]	[0; 1; 0]	[0; 0; 1]

## Data Availability

The data used to support the findings of this study are included within the article.
